# Arrhythmia Classification Algorithm Based on a Two-Dimensional Image and Modified EfficientNet

**DOI:** 10.1155/2022/8683855

**Published:** 2022-08-27

**Authors:** Cui-fang Zhao, Wan-yun Yao, Mei-juan Yi, Chao Wan, Yong-le Tian

**Affiliations:** College of Physics and Electronic Information Engineering, Zhejiang Normal University, Jinhua 321004, China

## Abstract

The classification and identification of arrhythmias using electrocardiogram (ECG) signals are of great practical significance in the early prevention and diagnosis of cardiovascular diseases. In this study, we propose an arrhythmia classification algorithm based on two-dimensional (2D) images and modified EfficientNet. First, we developed a method for converting original one-dimensional (1D) ECG signals into 2D image signals. In contrast with the existing classification method that uses only the time-domain features of a 1D ECG signal, the classification of 2D images can consider the spatiotemporal characteristics of the signal. Then, to better assign feature weights, we introduced an attention feature fusion module (AFF) into the EfficientNet network to replace the addition operation in the mobile inverted bottleneck convolution (MBConv) structure of the network. We selected EfficientNet for modification because, compared with most convolutional neural networks (CNNs), EfficientNet does not require manual adjustment of parameters, which improves the accuracy and speed of the network. Finally, we combined the 2D images and the improved EfficientNet network and tested its performance as an arrhythmia classification method. Our experimental results show that the network training of the proposed method requires less equipment and training time, and this method can effectively distinguish eight types of heartbeats in the MIT-BIH arrhythmia database, with a classification accuracy of 99.54%. Thus, the model has a good classification effect.

## 1. Introduction

The 2020 report on cardiovascular health and disease in China shows that the incidence and mortality of cardiovascular disease have been increasing, while the age of onset has been decreasing [1]. Arrhythmia is an important group of cardiovascular diseases, and its early detection plays a crucial role in the treatment of cardiovascular diseases. The diagnosis of arrhythmia mostly depends on the electrocardiogram (ECG), and the classification of arrhythmia by analyzing the ECG has become a hot research topic [2].

The traditional classification and identification of arrhythmia rely mainly on extracting features [3] such as timing features, statistical features, and morphological features [4–7]. The QRS complex, the most widely utilized feature in the field, is generally processed by employing Hermite polynomials, wavelet transforms, high-order statistics, and other techniques before extracting morphological characteristics [5–13]. Because of the emergence of deep learning, researchers often use neural network feature selection instead of manual feature selection to achieve automatic feature extraction [14–25]. Hannun et al. [19] directly input the one-dimensional (1D) ECG signal into the improved ResNet-34 deep learning network for the first time, realizing end-to-end arrhythmia classification. Lu et al. [24] used the convolution method to convert the 1D ECG signal into a two-dimensional (2D) image for the first time, and they fused temporal features for the classification of five types of arrhythmia, with an accuracy rate of 99%. Huang et al. [20] converted ECG signals into time-spectrograms through a short-time Fourier transform, and used 2D convolutional neural networks (CNNs) to classify five types of arrhythmias, achieving an accuracy of 99%. Compared with the 1D training accuracy of 90.93%, the 2D image training effect was better. Naz et al. [23] converted ECG signals into 32 × 32 binary images and used several deep CNNs for ventricular tachyarrhythmia recognition, achieving an accuracy of 97.6%. Maskeliunas et al. [25] obtained the statistical features extracted from 2D images based on Gramian angular field (GAF), achieving 86% accuracy in the classification of premature ventricular contraction (PVC) beats versus normal (NOR) beats. Akbar et al. [17] extracted ECG signal features based on time-spectral entropy and input them into the CNN, realizing the classification of five types of arrhythmias, and the classification accuracy reached 98.33%. In the same year, Min et al. [21] used the GAF transformation to convert 1D signals into 2D signals and then utilized the transfer CNN to achieve the classification of five types of arrhythmias. The above methods convert 1D ECG signals into 2D signals and use neural networks to classify them with good results, but manual parameter tuning is required in most CNN structures, the number of iterations is high, the process is complex and time-consuming, equipment requirements are high, there are few types of arrhythmias involved in arrhythmia classification, and there is still room to improve the classification accuracy.

To improve classification accuracy, the width, depth, or resolution of the network is generally increased. Although two or three dimensions can be arbitrarily scaled, arbitrary scaling requires tedious manual tuning, and usually still produces sub-optimal accuracy and efficiency. Tan et al. [26] proposed EfficientNet, whose main idea is to search for an efficient baseline and then use hybrid scaling, which combines depth, width, and resolution scaling according to certain rules. It has few network parameters and a much higher speed while providing good accuracy, which improves the practicality of the network as well as the industrial landing possibility. Through transfer learning, the EfficientNet network has achieved a good level of performance on several well-known data sets and good results in medicine [27–30]. Feature fusion is usually implemented with simple linear operations. Attention feature fusion (AFF) [31] can better fuse semantically inconsistent and scale-inconsistent features and is suitable for short connections.

In this study, we developed a preprocessing method to convert 1D ECG signals into 2D images and modified the EfficientNet network to achieve arrhythmia classification. We selected EfficientNet for modification due to its transfer learning capabilities, fast training speed, and high efficiency and because it does not require manual adjustment of network parameters. The aim of the modification was to improve EfficientNet and apply it to arrhythmia classification. The novelty and contribution of this study are as follows:

1. A preprocessing method is proposed to convert the original 1D ECG signal into a 2D image, which reflects the spatiotemporal features of the signal.
2. AFF is introduced to replace the addition operation in the MBConv structure of the EfficientNet network.
3. The proposed method effectively distinguishes eight types of heartbeats in the MIT-BIH arrhythmia database, with a classification accuracy of 99.54%.

## 2. Materials and Methods

In this section, we will briefly introduce the database that we used for ECG classification and describe our data preprocessing and network. The flow diagram of the proposed method is shown in Figure 1.

### 2.1. Database

We obtained the experimental data in this study from the MIT-BIH arrhythmia database, which has approximately 110,000 ECG beats, including 16 different types of arrhythmias [32, 33]. Considering that unclassifiable beats such as paced heartbeats in the database have usually been ignored in prior ECG arrhythmia classification studies, we selected eight common arrhythmias for classification in this study: NOR, PVC, paced beat (PAB), right bundle branch block beat (RBBB), left bundle branch block beat (LBBB), atrial premature contraction (APC), ventricular flutter wave (VFW), and ventricular escape beat (VEB). The selected data codes and sample numbers are shown in Table 1.

### 2.2. Preprocessing

ECG signal preprocessing mainly refers to beat segmentation and signal filtering. Generally, a relatively complete ECG signal includes at least the *P* wave, QRS complex, and T wave, and the time intervals of each waveband are shown in Table 2 [34]. It can be seen from Table 2 that the minimum duration of the complete *P* wave, QRS complex, and T wave is 0.44 s (including the *P*–*R* interval and *Q*–*T* interval). Combined with the sampling frequency of 360 Hz, a relatively complete heartbeat sequence length of at least 158 sample points can be obtained.  Figure 2(a) shows the original waveform of an ECG signal, whose horizontal coordinate is the number of sampling sequence points, and the vertical coordinate is the amplitude of the ECG signal. We took the *R*-peak marked by the expert as the dividing point and extended point *m*1 to the left (including the *R*-peak point), extended point *m*2 to the right (excluding the *R*-peak point), and performed dynamic segmentation to form a cardiac slice, which contained a relatively complete *P* wave, QRS complex, and *T* wave. Then, we made a single heartbeat ECG signal waveform diagram, setting *A*={*A*_1_, *A*_2_,……*A*_*t*_}, as shown in Figure 2(b), where the displayed abscissa range is [*n*_min_, *n*_max_], and the ordinate range is [*A*_min_, *A*_max_]. To unify the distribution of beats, we normalized the beats and converted them into 2D images. We set the amplitude of the ECG signal as {*Af*_*n*_, *n* ∈ [1, *m*1+*m*2]} and the pixel value of the 2D image as {*I*_*a*,*b*_, *a* ∈ [1,224], *b* ∈ [1,224]}. The corresponding point relationship of the conversion from the 1D ECG signal to the 2D image signal is shown in Figure 2(b), and the conversion formulas are as follows:

(1) $$\begin{array}{c} I\left(a,b\right)=\left\{\begin{array}{cc} 255*\frac{Af_{n}-min\left(Af_{n}\right)}{\max\left(Af_{n}\right)-\min\left(Af_{n}\right)} & a=x\&b=y\\ 255 & else \end{array}\right., \end{array}$$

(2) $$\begin{array}{c} x=224*\frac{n-n_{\text{min}}}{n_{\text{max}}-n_{\text{min}}}, \end{array}$$

(3) $$\begin{array}{c} y=224*\frac{Af_{\text{n}}-A_{\text{min}}}{A_{\text{max}}-A_{\text{min}}}. \end{array}$$

Among these formulas, (1) returns the pixel expressions for 2D images, (2) is the formula for transforming the horizontal coordinates of 2D images, and (3) is the formula for transforming the vertical coordinates of 2D images. The pseudocode of the proposed preprocessing method is shown in Algorithm 1.

There is a lot of noise in the process of ECG signal acquisition owing to the influence of the in vivo and in vitro environment; thus, we used the morphological corrosion function to denoise the 2D images to create a heartbeat sample.

## 3. Improved EfficientNet

EfficientNet features several distinct network models ranging from B0 to B7, with B1 to B7 continuously increasing the number of layers, parameters, and sub-blocks based on B0. Simultaneously, the resolution of the input image is growing, which means that equipment needs are continually increasing. Here, we chose the EfficientNet-B0 network as the classification model based on the features included in the 2D images of the cardiac slices and the hardware resources of the available equipment. The network input image resolution requirement for EfficientNet-B0 is 224 × 224. As shown in the analysis in Section 2.2, transforming the waveform picture into an image with a resolution of 224 × 224 meets the requirements.

The MBConv module is the core structure of the EfficientNet-B0 network. Its structural diagram is shown in Figure 3(a). A simple addition operation is used to realize the feature fusion of different branches. In this study, we introduced the AFF [31] to replace the addition operation in the MBConv structure so as to better allocate the weight of the features. The improved MBConv structure is shown in Figure 3(b), and the mapping relationship of AFF is

(4) $$\begin{array}{c} Z=M\left(X\cup Y\right)⊗X+\left(1-M\left(X\cup Y\right)\right)⊗Y, \end{array}$$

where ∪ is the initial feature fusion of the two input features (*X* and *Y*), *M* is the multi-scale attention module function, and ⊗ represents feature multiplication.

## 4. Results and Analysis

To validate the effectiveness of the algorithm, we performed model training on Intel CPU, NVIDIA GTX1650 GPU, using the Python-based PyTorch framework with PyTorch 1.9 and Python 3.8. We randomly divided the ECG signal image data set into two parts: the training set of 96,858 images, 20% of which we designated as the validation set (19,371 images), and the test set of 10,762 images.

### 4.1. Heartbeat Sequence Length Comparison Experiment

From Section 2.2, we know that a more complete heartbeat sequence containing a complete *P* wave, QRS complex, and *T* wave is at least 158 sample points in length. When the intercepted heartbeat sequence is too short, the sample will contain insufficient information, and the classification accuracy will be low; when the sequence is too long, the sample will contain a large amount of information, but some information may be redundant, so there is little room for improving the classification accuracy, and the time it takes to initialize data increases.

In this study, we used varied sequence lengths (*L*) for related experiments to verify the influence of heartbeat sequence length on classification performance. We defined *L* as 130, 160, 170, 180, 190, 200, and 250 sample points, with corresponding left and right extension points (*m*1 and *m*2) satisfying *m*1 = *m*2 = 65, *m*1 = *m*2 = 80, *m*1 = *m*2 = 85, *m*1 = *m*2 = 90, *m*1 = *m*2 = 95, *m*1 = *m*2 = 100, and *m*1 = 100 and *m*2 = 150, respectively.  Figure 4(a) depicts the accuracy of the training set versus the number of epochs of model training for the different sequence lengths. The accuracy of the training set under different sequence lengths is largely stable after 300 epochs. We chose the best model for testing, and Figure 4(b) shows the accuracy comparison graph of the test set over various lengths. As *L* increases, the accuracy of the test set increases from 130, peaks at 180, and then declines. This suggests that the duration of the heartbeat sequence influences accuracy and different sequence lengths contain varied ECG signal properties. Although the physical properties of the QRS complex are the most important for defining the heart rate type, the *P* wave and *T* wave also have an impact on the classification outcomes. *L* = 130 contains mostly the QRS complex and has an incomplete *P* wave and *T* wave; *L* = 160–200 includes a more complete *P* wave, QRS complex, and *T* wave with more features; and *L* = 250 includes not only a complete *P* wave, QRS complex, and *T* wave but also a gentle wave before and after the *P* wave and after the *T* wave. Too many sample points make features less distinct while also causing accuracy swings. Additionally, as seen in Figure 4(c), more sample points equate to a longer training time.

Considering the inevitable data imbalance in the medical data set sample, we employed evaluation metrics such as sensitivity, specificity, and precision [20] for further comparison, with the results displayed in Figure 5. When comparing the evaluation indexes in Figure 5, it can be seen that the total index of *L* = 180 is better than that of other examples, particularly in APC, where the precision rate and sensitivity are greatly increased. The type of arrhythmia is more accurate in general.

### 4.2. Experiment on Classification of EfficientNet Network before and after Improvement

To verify the performance of the classification method based on the improved EfficientNet network, we conducted experiments on a sample library of heartbeats with a sequence length *L* = 180. To ameliorate the data imbalance problem in the medical data set samples, we performed data augmentation for two types of samples: VEB and VFW; we added four data sets with the heartbeat sequence lengths *L* = 160, *L* = 170, *L* = 190, and *L* = 200 to the data set of *L* = 180.

Table 3 shows the outcomes of EfficientNet before and after improvement, as well as the classification evaluation indexes before and after data augmentation. Compared with other methods, AFF-EfficientNet-B0 + data augmentation has significantly higher accuracy for APC and VFW compared to the other three methods, with an overall accuracy of 99.54. APC is a common clinical arrhythmia with symptoms such as palpitations, and some people may be asymptomatic; VFW is more commonly observed in those with serious heart problems and is diagnosed mostly through an ECG examination. Thus, the results indicate that the revised model enhances APC and VFW recognition accuracy and makes follow-up treatment easier.

The classification confusion matrix of AFF-EfficientNet-B0 + data augmentation is given in Figure 6. Figure 6 shows that the categorization accuracy of all eight ECG signal types is relatively high, and there is relatively more confusion between the three categories of APC, PVC, and NOR.

Figure 7 shows the typical correct sample heartbeat maps, and Figure 8 shows some of the misidentified sample heartbeat maps. The main reason for the misclassification of APC as NOR in Figure 8(a) is that this APC heartbeat picture has a large difference at the *P* wave compared to most of the samples in the APC library, and the reason for the misclassification of NOR as APC in Figure 8(b) is that in addition to the *P* wave, there is also a large undulation at its *T* wave, which is different from the normal NOR sample in Figure 7.

In addition, the heartbeat of the same patient generally has the greatest similarity in terms of APC and NOR; for example, patient number 100 was recorded to have both APC and NOR, so this also contributed to some extent to the result that the model sometimes confused APC and NOR. In Figure 8(c), the NOR sample mistakenly detected as a PVC sample was similar to the normal PVC sample in Figure 7, which was an atypical case in the NOR sample pool. The same was true for the PVC sample misclassified as a NOR sample in Figure 8(d).

The analysis of the classification accuracy by sequence length and the analysis of the misclassified samples indicate there are obvious shortcomings in existing methods that use the QRS complex as the main feature for ECG signal classification, and the small undulations on both sides of the QRS complex have some influence on the classification accuracy. Thus, the classification based solely on the QRS complex is not ideal.

### 4.3. Comparison Experiments with Other Classification Algorithms

Table 4 shows the results of comparing the algorithm in this paper with other algorithms, all using the MIT-BIH arrhythmia database. Plawiak and Acharya [35] used 10 s as the time base to intercept ECG signal samples to build a database, employed the discrete Fourier transform to extract features, and combined the features with the CNN for classification and identification. With a small number of classification samples, the accuracy reached 95%. Liu et al. [35] used heartbeats from a database established by baseline intercepted samples and extracted the signal features under eight different time windows using a wavelet scattering transform. After using principal component analysis (PCA) for dimensionality reduction and a *k*-nearest neighbor classifier for four classifications, they obtained an accuracy of 99.3%. Yang et al. [15] extracted ECG morphological parameters, such as amplitude, time interval, and QRS complex morphological features and combined them with the *k*-nearest neighbor classifier for 15 classifications, achieving an accuracy of 97.7%. Romdhane et al. [36] used the focal loss to construct a novel loss function and optimized the CNN model to achieve five end-to-end classifications with an accuracy of 98.41%. Several recent papers have the problem of data imbalance, which is the norm for medical data sets.

In this study, eight categories of classification were achieved, with an accuracy of 99.54%, which was higher than the accuracy of existing arrhythmia classification methods, but the same problem of sample imbalance existed; increasing samples and evaluation metrics such as specificity and sensitivity were used to mitigate this problem. In comparison to existing methods, the accuracy of the method proposed in this study was found to be higher, and it achieved the classification of more categories. In addition, the proposed method had low equipment requirements and fast training and testing time. The average training time for each epoch was 4.5 min; the single test time was 0.0027 s; and the model size was 16,713 KB.

## 5. Discussion and Conclusion

In this study, we developed a method for converting original 1D ECG signals into 2D image signals. To better assign feature weights, we introduced AFF to replace the addition operation in the MBConv structure of the EfficientNet network.

The main limitation of the proposed arrhythmia classification algorithm is the low positive prediction accuracy for identifying APC beats. This is caused by data imbalance: specifically, there are many more NOR beats than other beats. The ratio of APC beats is only 2.3% in the data set. Moreover, multiple ECG samples from the same patient will generally exhibit the greatest similarity in heartbeats. The study results of the data augmentation show that the positive prediction accuracy for identifying VEB is substantially increased and ranges from 97.9% to 99.1%.

Given the influence of available laboratory equipment, we converted 1D ECG signals into 2D image signals and used spatiotemporal characteristics to perform classification experiments on eight ECG signal types in the MIT-BIH arrhythmia database, achieving relatively high accuracy of 99.54% based on the improved EfficientNet-B0 network. Most medical data sets have sample imbalance problems, which are generally mitigated by increasing a few types of samples or decreasing most types of samples. In this study, we applied the preprocessing method of 1D to 2D ECG signal conversion, which increased the amount of data, and selected the best length. Additionally, we performed data augmentation for two categories, VEB and VFW, and we added four similar groups of different-length images to this data set, which alleviated the data imbalance problem to some extent. Finally, we employed three evaluation indices, namely, sensitivity, specificity, and precision rate ground, to evaluate the model's effect, all of which were found to be high, indicating that the model has a good classification effect.

To extend the sample, the next step will be to identify relevant volunteers for sample collection. Validation of more ECG signal databases will be considered in the future to improve the practicality and robustness of the classification method for eventual application on medical robots or ECG signal monitoring devices. This approach can help doctors more accurately and quickly diagnose cardiovascular diseases from ECG signals [37].

## Figures and Tables

**Figure 1:** Flow diagram of the proposed method.

**Figure 2:** Data preprocessing: (a) heartbeat interception: extract a heartbeat from the original signal and (b) 1D to 2D: transform a 1D signal into a 2D image.

**Figure 3:** Comparison before and after the improvement of the MBConv structure: (a) the structure of MBConv and (b) the improved structure of MBConv, wherein AFF replaces the addition operation in the MBConv structure.

**Figure 4:** Comparison of accuracy for different heartbeat sequence lengths (*L*): (a) comparison of training set accuracy corresponding to different heartbeat sequence lengths, (b) comparison of test set accuracy corresponding to different heartbeat sequence lengths, and (c) comparison of training time corresponding to different heartbeat sequence lengths.

**Figure 5:** Comparison of test results for different heartbeat sequence lengths (*L*): (a) comparison of test sensitivity corresponding to different heartbeat sequence lengths, (b) comparison of test specificity corresponding to different heartbeat sequence lengths, and (c) comparison of test precision corresponding to different heartbeat sequence lengths.

**Figure 6:** Confusion matrix representation of the test classification results for *L* = 180.

**Figure 7:** Typical correct sample heartbeat maps. (a) NOR. (b) APC. (c) PVC.

**Figure 8:** Some misclassified sample heartbeat maps: (a) heartbeat images misclassified as NOR instead of APC, (b) heartbeat images misclassified as APC instead of NOR, (c) heartbeat images misclassified as PVC instead of NOR, and (d) heartbeat images misclassified as NOR instead of PVC.

**Algorithm 1:** Pseudocode of proposed preprocessing method.

**Table 1:** MIT-BIH arrhythmia database.

Type	Records	Number of beats
NOR	100, 101, 103, 105, 108, 112, 113, 114, 115, 117, 121, 122, 123, 202, 205, 219, 230, 234	75,016
PVC	106, 116, 119, 200, 201, 203, 208, 210, 213, 215, 221, 228, 233	7,130
PAB	102, 104, 107, 217	7,024
RBBB	118, 124, 212, 231	7,256
LBBB	109, 111, 207, 213	8,072
APC	209, 220, 222, 223, 232	2,544
VFW	207	472
VEB	207	106
**Total**		**107,620**

**Table 2:** Time interval table of each waveband of the ECG signal.

Wave	*P*	*P*−*R*	QRS	*Q*−*T*	*T*
Time interval (s)	0.12	0.12–0.20	0.06–0.10	0.32–0.44	0.05–0.25

**Table 3:** Comparison of sensitivity, specificity, and precision at *L* = 180.

Evaluation indicator	Method	Type							
		APC	LBBB	NOR	PAB	PVC	RBBB	VEB	VFW
Sensitivity	Method 1	0.89	0.995	0.998	1	0.989	0.997	1	0.979
	Method 2	0.906	0.996	0.998	1	0.99	0.999	1	0.987
	Method 3	0.909	0.998	0.998	1	0.989	0.997	1	0.979
	Method 4	0.902	0.998	0.999	1	0.987	0.997	1	0.991
Specificity	Method 1	0.89	0.995	0.998	1	0.989	0.997	1	0.979
	Method 2	0.906	0.996	0.998	1	0.99	0.999	1	0.987
	Method 3	0.909	0.998	0.998	1	0.989	0.997	1	0.979
	Method 4	0.902	0.998	0.999	1	0.987	0.997	1	0.991
Precision	Method 1	0.954	1	0.996	1	0.99	0.994	1	0.958
	Method 2	0.962	1	0.997	1	0.986	0.993	1	0.979
	Method 3	0.967	1	0.996	1	0.989	0.994	1	0.939
	Method 4	0.974	1	0.996	1	0.989	0.993	1	0.987

Notes: Method 1, Method 2, Method 3, and Method 4 represent EfficientNet-B0, EfficientNet-B0 + data augmentation, AFF-EfficientNet-B0, and AFF-EfficientNet-B0 + data augmentation, respectively.

**Table 4:** Comparison of different methods.

Author	Method	Type	Accuracy (%)	Number of samples
Plawiak and Acharya [35]	Welch method and discrete Fourier transform	17	95.00	744
Liu et al. [35]	Wavelet scattering transform	4	99.30	100,507
Yang et al. [15]	ECG morphological parameters and visual pattern characteristics	15	97.70	104,986
Romdhane et al. [36]	Building a deep CNN model	5	98.41	109,446
This paper	1D to 2D + AFF-EfficientNet	8	99.54	107,620

## Data Availability

Publicly available data sets were analyzed in this study. These data sets can be found at https://archive.physionet.org/physiobank/database/html/mitdbdir/mitdbdir.htm.
